The article "Dynamics in the Cytoadherence Phenotypes of Plasmodium falciparum Infected Erythrocytes Isolated during Pregnancy" was published in 2014. Journal: PLoS One.

# Dynamics in the Cytoadherence Phenotypes of *Plasmodium falciparum* Infected Erythrocytes Isolated during Pregnancy

**DOI:** 10.1371/journal.pone.0098577

**Published:** 2014-06-06

**Authors:** Justin Doritchamou, Sylvain Sossou-tchatcha, Gilles Cottrell, Azizath Moussiliou, Christophe Hounton Houngbeme, Achille Massougbodji, Philippe Deloron, Nicaise Tuikue Ndam

**Affiliations:** 1 PRES Sorbonne Paris Cité, Faculté de Pharmacie, Université Paris Descartes, Paris, France; 2 UMR216 Mère et enfant face aux infections tropicales, Institut de Recherche pour le Développement, Paris, France; 3 Centre d'Etude et de Recherche sur le paludisme associé à la Grossesse et à l'Enfance, Université d'Abomey-Calavi, Cotonou, Benin; 4 ED Physiologie Physiopathologie et thérapeutique Sorbone Université, Université Pierre Marie Curie, Paris, France; 5 Hôpital de zone de Suru Lere, Cotonou, Benin; University of Copenhagen, Denmark

## Abstract

Pregnant women become susceptible to malaria infection despite their acquired immunity to this disease from childhood. The placental sequestration of *Plasmodium falciparum* infected erythrocytes (IE) is the major feature of malaria during pregnancy, due to ability of these parasites to bind chondroitin sulfate A (CSA) in the placenta through the VAR2CSA protein that parasites express on the surface of IE. We collected parasites at different times of pregnancy and investigated the adhesion pattern of freshly collected isolates on the three well described host receptors (CSPG, CD36 and ICAM-1). *V*ar genes transcription profile and VAR2CSA surface-expression were assessed in these isolates. Although adhesion of IE to CD36 and ICAM-1 was observed in some isolates, CSA-adhesion was the predominant binding feature in all isolates analyzed. Co-existence in the peripheral blood of several adhesion phenotypes in early pregnancy isolates was observed, a diversity that gradually tightens with gestational age in favour of the CSA-adhesion phenotype. Infections occurring in primigravidae were often by parasites that adhered more to CSA than those from multigravidae. Data from this study further emphasize the specificity of CSA adhesion and VAR2CSA expression by parasites responsible for pregnancy malaria, while drawing attention to the phenotypic complexity of infections occurring early in pregnancy as well as in multigravidae.

## Introduction

Despite the substantial protective anti-malarial immunity gradually acquired during childhood in residents of areas with high malaria transmission, during their first pregnancy women are more at risk of infection by *Plasmodium falciparum* compared to non-pregnant adults [1]. The sequestration of *P. falciparum*-infected erythrocytes (IE) in the placenta is the key characteristic of pregnancy-associated malaria (PAM), and can be associated with intense inflammatory activity. The latter is more common in women during their first pregnancy. The pregnancy-specific aspect has been attributed to parasites expressing particular variant surface antigens [2], [3]. Severe maternal anemia and delivery of babies with low birth weight are the major consequences associated with the accumulation of IE in the placenta [4]. The best-characterized adhesion ligands expressed on the surface of IE are members of the highly polymorphic *Plasmodium falciparum* erythrocyte membrane protein-1 (PfEMP-1) family, encoded by the *var* gene family [5]. *Var* genes can be classified into 5 majors groups (A to E) based on the sequence polymorphism observed both in the non-coding upstream region and also in the coding sequence [2], [6]–[8]. A particular PfEMP1, named VAR2CSA, is now recognized as the main parasite ligand mediating IE binding to placental tissue [2], [9], [10].

The article "Dynamics in the Cytoadherence Phenotypes of Plasmodium falciparum Infected Erythrocytes Isolated during Pregnancy" was published in 2014. Journal: PLoS One.

Numerous characteristics of VAR2CSA make it the major candidate for development of a vaccine to prevent PAM, characteristics that have been described in multiple studies [2], [9], [11]–[19]. However, data concerning the adhesion patterns of parasite isolates collected throughout pregnancy, and the kind of interactions that can characterize isolates present at different times of pregnancy, remain fully to be generated. Although it has been suggested that other molecules (hyaluronic acid and non-immune globulins) may participate in the adhesion of IE in the placenta [20]–[22], several lines of evidence indicate that CSA is the most important receptor involved [2], [3], [17], [23]–[28]. Endothelial receptors, such as CD36 and ICAM-1, commonly support the adhesion of field isolates [26] from non-pregnant patients [29]–[31]. However, it has been shown that these two receptors are highly expressed in the placenta and ICAM-1 has been localized on syncytiotrophoblasts, suggesting a possible role in the placental sequestration of IE [32]. Other studies have nevertheless reported that placental isolates do not bind to CD36 [20], [22] and ICAM-1 [25]. Thus, the function and the level of involvement of these molecules in the binding ability of IE collected from cases of PAM are still not well explored. In this study, we sought to characterize the binding properties *ex vivo* of field isolates collected from pregnant women at different time-points of pregnancy using three receptors expressed in the placenta that are known to support IE binding (CSPG, CD36 and ICAM-1). In addition, we investigated whether other pregnancy-related factors influence the parasite adhesion properties and whether infection by parasites with a particular adhesion pattern could be associated with poor pregnancy outcomes.

The article "Dynamics in the Cytoadherence Phenotypes of Plasmodium falciparum Infected Erythrocytes Isolated during Pregnancy" was published in 2014. Journal: PLoS One.

## Material and Methods

### Study design, collection and handling of blood samples

Written informed consent was given by all women participating in this study. The study was approved by the ethics committee of the Faculty of Health Science (University of Abomey-Calavi) in Benin. The study was conducted at the Suru Léré maternity clinic, Cotonou, Benin. All women were tested for *P. falciparum* infection using a rapid diagnostic test (Parascreen, Zephyr Biomedicals Goa, India), and those with a positive result were included. *P. falciparum* IE were obtained from 123 pregnant women attending antenatal visit and 9 women admitted for delivery. Venous blood was collected in vacutainers with citrate phosphate dextrose adenine anticoagulant. Thick and thin blood films were prepared from blood samples to confirm *P. falciparum* infection. Hemoglobin values of women and the birth weight of their offspring were collected for all women included at delivery. Detailed characteristics of the study site have been previously described [33].

Ring stage IE were allowed to mature *in vitro* to trophozoite-stage, as described [34]. Briefly, isolates were grown in RPMI 1640 supplemented with Hepes and L-glutamine (Lonza Biowhittaker), 0.3 g/L l-glutamine, 0.05 g/L gentamicin, 5 g/L albumax. Cultures were grown for no more than 48 h before testing. Ring stage parasites were also conserved in 10 volumes of TRIzol reagent (Invitrogen) and stored at −80°C until RNA extraction.

### Flow cytometry and binding assays

VAR2CSA expression on the surface of *P. falciparum* IE was assessed by flow cytometry using specific anti-VAR2CSA IgG as previously described [35]. Briefly, 2×10^5^ late-stage IE enriched by filtration on a magnetic column (VarioMACS, Miltenyi) were labelled with ethidium bromide, and sequentially exposed to anti-VAR2CSA rabbit IgG (final concentration 10 µg/ml), and to FITC-conjugated anti-rabbit IgG (1.5 mg/ml, Invitrogen). The anti-VAR2CSA rabbit IgG were purified from the plasma of rabbits previously immunized with the extracellular full-length protein from FCR3 strain [33]. A FACSCalibur flow-cytometer (BD Biosciences) was used to acquire the data, and the median fluorescence intensity (MFI) was determined. VAR2CSA surface expression was considered positive with an MFI ratio (MFI with IgG from rabbits immunized with VAR2CSA/MFI with IgG from rabbits before immunization) >1.2, as previously described [35].

A static assay that measures the adhesion to purified, immobilized receptors was used to assess the binding patterns of isolates, as described [36]. Briefly, 5 µg/ml of CSPG-Decorin (Sigma) or 10 µg/ml of ICAM-1 (R&D Systems) or CD36 (R&D Systems) or bovine serum albumin (Sigma) were diluted in PBS, and coated as spots in a 100×15 mm Petri dish (Falcon 351029). Late-stage IE enriched on a magnetic column (VarioMACS, Miltenyi), with a parasite density adjusted to 20% in 1×10^5^ cells were blocked in BSA/RPMI for 30 minutes at room temperature (RT), and allowed to bind to coated receptors for 15 minutes at RT. Unbound cells were removed by an automated washing system. Bound IE were fixed with 1.5% glutaraldehyde in PBS, stained with Giemsa, and quantified by microscopy, as the number of IE bound per mm^2^. Each sample was performed in duplicate. Based on the binding level of IE observed on BSA spots (data not shown), a threshold of significant adhesion was determined as the mean +3 standard deviations and was set as binding ≥35 IE/mm^2^.

The article "Dynamics in the Cytoadherence Phenotypes of Plasmodium falciparum Infected Erythrocytes Isolated during Pregnancy" was published in 2014. Journal: PLoS One.

### RNA extraction, cDNA synthesis and quantification of var gene transcripts

Thawed samples stored in TRIzol reagent were used to extract the total RNA, as recommended by the manufacturer. The dried pellet was resuspended with 10 µl of DEPC-water. RNA samples were treated with DNase I (Invitrogen) for 30 min at RT. The absence of gDNA in RNA samples was confirmed by no parasite DNA amplification after 40 cycles of real-time PCR performed with *seryl-tRNA synthetase P. falciparum*-specific primers, using a Rotorgene 6000 thermal cycler system (Corbett Research). Reverse transcription of DNA-free RNA was performed using Thermoscript (Invitrogen) with random hexamer primers in a total volume of 20 µl, as recommended by the manufacturer.

*Var* gene transcripts abundance was quantified by qPCR, as described [36]. Briefly, runs were performed (95°C for 1 min, followed by 40 cycles of 94°C for 30 s, 54°C for 40 s, and 68°C for 50 s) in a final volume of 20 µl, using 0.5 µl cDNA; 1×SYBR Green Mastermix (Bioline) and 1.25 µM of specific primer pairs for individual gene or *var* gene subtypes. Primer pairs targeting the conserved region of *var2csa* [9] and previously designed specific *var*-type primers (A1, B1, B2, C1, C2, *var1*, and *var3*) were used, as described [37]. *Seryl-tRNA synthetase* (primer pair p90) and *fructose-bisphosphate aldolase* (primer pair p61) were used as endogenous controls [2]. Non-template controls and the 3D7 gDNA, used as calibrator, were performed for validation on every run. The melting curve analysis was done to ensure the amplification specificity. Samples with Cycle Threshold (CT) values exceeding 35 were not quantified. The relative copy number of *var* genes transcripts was determined, as described [36].

The article "Dynamics in the Cytoadherence Phenotypes of Plasmodium falciparum Infected Erythrocytes Isolated during Pregnancy" was published in 2014. Journal: PLoS One.

### Statistical analysis

Statistical analysis was performed using STATA software version 11 (Stata corporation, College Station, Texas, United States) and data were plotted using Prism software (version 5, Graph-Pad). Transcripts with abundance values greater than 5% of the total *var* genes analyzed were listed. Continuous variables were compared by the Mann-Whitney and Kruskall-Wallis tests. The Wilcoxon matched pairs test was used to compare matched variables. A linear regression model was used to analyze the binding level of parasites to each host receptor according to the parity of women, the timing of pregnancy and surface expression of VAR2CSA. The same analysis was performed on the data defined as positive and negative binding to each receptor using a logistic regression model. This latter model was performed, in addition to linear model, to describe and predict the binding pattern of isolates that infect women throughout pregnancy in relation with the parity status of these women.

## Results

### Transcription profile of var genes by isolates collected from pregnant women

Parasites were obtained from 132 pregnant women with a *P. falciparum* infection, as confirmed by microscopical examination. The clinical characteristics of these women are presented in Table 1. Analysis of *var* genes transcripts diversity was performed on 100 cDNA successfully synthesized. Although transcripts of several *var* genes were detected in most of the isolates, transcript of *var2csa* was detected in 99 out of the 100 tested cDNA. Isolates highly transcribed *var2csa* compared to other *var* genes (*P<0.0001*, Figure 1). The median copy number of *var2csa* detected among these isolates was 6.8 (IQR, 1.8–19.0) whereas other *var* genes coverage by specific primers targeting A1, B1, B2, C1, C2, *var1* and *var3* showed a median copy number <0.2. Moreover, *var1* was exclusively transcribed by one isolate (OPT173), and transcripts of *var2csa* were exclusively detected in eight isolates.

**Table 1:** Clinical characteristics of the women and their offspring birth weight.

N = 132	Mean	Median	IQR
Parasitemia (/µl)	71,781	18,207	3,927–59,719
Age (years)	26.3	27	21–30
Parity	2.9	2	1–4
Gestational age (weeks)	22	23	12–28
Hemoglobin (g/dl)	9.6	9.7	8.8–10.6
Birth weight of the offspring (g)	3017	3000	2750–3350

### Adhesion phenotype of field isolates from pregnant women

To limit changes in the structure of parasite populations in the isolates studied, the culture time required *in vitro* to obtain mature stages used in the binding phenotyping was limited to 48h. Isolates with very low parasite density that required longer cultivation time to yield sufficient IE were not retained for analyses. The ability of parasites isolated from pregnant women to bind to host receptors (CSPG, CD36, and ICAM-1) was assessed on 54 successfully-matured isolates (50 samples collected during pregnancy and 4 samples obtained at delivery). Among these women, 13 were primigravidae and 41 were multigravidae. The levels of binding to each receptor (CSPG, CD36, and ICAM-1) are shown in Table 2. Distinct binding ability was observed among the parasite isolates. Although binding intensity also differed according to receptors, most of the tested isolates showed adhesion to at least one of the receptors (Table 2). Five isolates were not tested on CD36 and ICAM-1 due to limited amounts of IE. However, significant adhesion to CSPG was observed on 32 (59.2%) isolates, whereas 13 (26.5%) and 2 (4.1%) isolates showed substantial levels of binding to CD36 and ICAM-1, respectively (Figure 2A). Overall, isolates bound at significantly higher levels to CSPG (median  = 81.5, 14.7–320.5) than to CD36 (8.0, 0–39.5) (*P = 0.001*) and to ICAM-1 (0, 0.0–5.5) (*P<0.0001*). Furthermore, the binding intensity to ICAM-1 was also lower than to CD36 (*P = 0.0004*), suggesting that affinity to this receptor may of less importance to isolates from pregnant women.

The article "Dynamics in the Cytoadherence Phenotypes of Plasmodium falciparum Infected Erythrocytes Isolated during Pregnancy" was published in 2014. Journal: PLoS One.

**Figure 1:** Transcription level of *var* genes were shown as relative copy number. Bars indicate the median of distribution.

**Table 2:** *Var* genes transcription profile and adhesion phenotype of 54 isolates collected from pregnant women in Cotonou, Benin.

Isolates	Dominant *var* gene(s) transcribed	Transcripts relative abundance (% of total *var*)	MOI	VAR2CSA surface detection	CSPG	CD36	ICAM-1
OPT079	*var2csa; upsC*	92; 6	2	1.2	41	nd	nd
OPT081	*upsB; upsA; upsC*	46; 31; 11	5	0	12	917	0
OPT091	*upsB; var1; upsA*	58; 26; 8	1	1.4	13	nd	nd
OPT101	*var2csa; upsC*	61; 39	4	1.2	28	nd	nd
OPT105	*var2csa*	99	4	2.7	255	nd	nd
OPT106	*var2csa; upsC; upsA*	71; 12; 10	4	1.2	148	nd	nd
OPT107	*var1; upsB; upsC; var2csa*	39; 29; 24; 7	3	1	8	903	0
OPT109	*var2csa*	99	5	2.3	275	21	17
OPT110	*var2csa*	98	6	1.4	261	13	0
OPT114	*var2csa*	98	2	2.4	0	5	0
OPT115	*var1; upsC; var2csa,*	49; 32; 17	1	1	7	111	64
OPT116	*var2csa; var3*	77; 23	1	2.4	15	39	0
OPT118	*var2csa*	99	4	3.6	250	0	0
OPT119	*var2csa; upsC; upsA*	50; 43; 6	2	3.3	10	19	12
OPT120	*var2csa; var1*	86; 9	3	1.5	14	414	6
OPT124	*var2csa*	94	1	3	87	65	0
OPT127	*var2csa; var1*	92; 5	1	3.4	446	14	0
OPT130	*var1; upsB; upsA*	70; 21; 7	4	4.1	746	6	9
OPT133	*upsC; var1; upsA; var2csa*	52; 17; 16; 8	1	0.9	7	175	32
OPT135	*var1; upsB; upsA; upsC; var2csa*	29; 24; 21; 18; 7	1	1	18	483	14
OPT137	*var2csa*	99	1	1.6	37	0	0
OPT139	*var2csa; upsB*	85; 6	3	1.5	6	32	0
OPT140	*var2csa*	98	4	1.6	253	8	0
OPT141	*var2csa*	99	3	3.7	492	6	0
OPT144	*var2csa*	97	3	3	414	8	0
OPT145	*upsC; var1; var2csa; upsA; var3*	29; 25; 19; 16; 6	2	1	10	28	0
OPT148	*var2csa; var1; upsC*	81; 7; 7	4	2	31	22	0
OPT151	*var2csa; upsC*	91; 7	4	3	715	0	0
OPT154	*var2csa; var1*	93; 5	2	3.4	632	0	0
OPT158	*var2csa; var1*	91; 7	2	1.9	108	0	0
OPT161	*var2csa*	98	4	2.5	401	0	0
OPT165	*var2csa; var1; upsB, upsC*	35; 31; 23; 8	2	0.8	5	0	9
OPT166	*var2csa*	97	4	1.6	41	0	0
OPT169	*var2ca*	98	1	6.7	263	0	0
OPT173	*var1*	100	1	0.3	0	91	0
OPT175	*upsC; var2csa*	75; 20	3	0.8	27	65	6
OPT178	*var2csa*	98	2	2.6	54	0	14
OPT180	*var2csa; upsC*	93; 5	7	4	314	0	0
OPT184	*upsA; upsB*	57; 36	1	1.2	26	8	0
OPT220	*var2csa*	100	1	2.4	277	11	2
OPT225	*var2csa; uspA*	71; 28	3	1.9	136	29	1
OPT246	*var2csa; var1; upsA*	65; 22; 10	5	3.2	600	14	1
OPT248	*var2csa; uspC*	81; 18	3	2.9	126	40	5
OPT252	*var1; var2csa*	58; 40	4	1.8	340	107	4
OPT262	*var2csa; var1*	75; 18	5	3.8	509	5	1
OPT266	*var2csa; var1*	77; 20	3	1	183	7	4
OPT267	*var1; var2csa; upsA, upsC*	69; 13; 9; 6	3	4.3	354	13	4
OPT270	*var1; var2csa; upsB*	47; 43; 5	4	0.6	32	4	46
OPT272	*var1; var2csa; upsA*	52; 39; 5	5	0.8	15	44	23
PAM04	*var2csa*	96	1	2	28	0	0
PAM05	*var1*	94	2	2.5	76	0	0
PAM06	*var2csa*	99	1	7.6	0	5	0
PAM07	*var2csa*	97	1	3.1	1256	0	0
PAM08	*var2csa*	99	7	2.9	964	0	0

Transcription data are presented as the relative abundance of the total *var* studied. Only transcripts whose levels were greater than 5% of all transcripts detected are listed. Binding data corresponding to each receptor are expressed as the number of bound infected erythrocytes per mm^2^ (IE/mm^2^).

The article "Dynamics in the Cytoadherence Phenotypes of Plasmodium falciparum Infected Erythrocytes Isolated during Pregnancy" was published in 2014. Journal: PLoS One.

**Figure 2:** Adhesion profile of isolates from pregnant women. The binding phenotype of isolates was assessed on CSPG, CD36 and ICAM-1 receptors and presented as proportion of “positive” adhesion to each receptor, defined at binding ≥35 IE/mm^2^ (A) – The binding profile of all tested isolates and (B) The segregation of the isolates binding profile according to the parity of women.

### Relationship between VAR2CSA expression and the CSA-binding phenotype

*Var2csa* is the only gene among the *var* genes examined in this study that was detected in all of the 54 successfully-matured isolates. To further refine the analysis we focus on the dominant transcripts detected. Only *var* genes with transcript abundances greater than 5% of the total *var* gene transcription [38], are reported in Table 2 and the most prevalent transcript indicates the dominant *var* gene of each isolate. Transcript abundance of *var2csa* above the threshold (5%) was observed in 48 out of 54 isolates whereas transcripts of *var1* and group ABC *var* genes were observed in 22/54 and in 25/54 (13/54 for *var* group A; 9/54 for *var* group B and 17/54 for *var* group C) of isolates, respectively (Table 2). *Var2csa* was exclusively or dominantly transcribed by 36 isolates. *Var1* was dominantly transcribed by 10 isolates, while *var* genes from groups ABC were dominantly transcribed by 6 isolates. The distribution of the transcription levels of the three categories of *var* genes (*var1*, *var2csa* and *var* ABC) was different in the two groups of parasite phenotypes (Fisher Exact Test; *P<0.0001*). Transcripts of *var1* was the predominant transcript detected (46%) among isolates with a CD36-binding phenotype (Table 3) while *var2csa* was (87%) in isolates binding to CSPG.

The article "Dynamics in the Cytoadherence Phenotypes of Plasmodium falciparum Infected Erythrocytes Isolated during Pregnancy" was published in 2014. Journal: PLoS One.

**Table 3:** Predominant *var* genes transcripts in PAM isolates adhering to CSA and CD36, *P<0.0001* *.

*var* gene groups	*var ABC*	*var1*	*var2csa*
CSA-adhering isolates^a^ (n = 32)	0	12.5	87.5
CD36-adhering isolates^a^ (n = 13)	23	46	31

*Fisher Exact test.

a adhesion defined as binding ≥35 IE/mm^2^.

Transcription data and that of VAR2CSA expression on the surface of IE were further analyzed in relation to the adhesion properties of the isolates (Table 4). Among the 32 isolates that showed significant binding to CSPG, significant labeling of the IE surface by anti-VAR2CSA antibodies was observed while only one isolate (OPT091) was recognized among isolates which did not show a CSPG binding phenotype (*P = 0.005*). Although all these CSA-adhering isolates transcribed *var2csa*, only 28 (87.5%) transcribed it as the dominant *var*. Among the 22 isolates which did not significantly bind to CSPG, *var2csa* was dominantly transcribed in 10 (45.4%), all of which were labeled by VAR2CSA antibodies. In five isolates a positive surface labeling was observed despite the fact *var2csa* was not the predominant transcript or just hardly detected.

**Table 4:** CSA-binding isolates and VAR2CSA surface expression in PAM isolates predominantly transcribing *var2csa* and non-*var2csa* genes.

Dominant *var* gene transcribed	CSA-adhering isolates^a^ (n = 32)	VAR2CSA surface detection**	Non or weakly CSA-adhering isolates^b^ (n = 22)	VAR2CSA surface detection**
*var2csa*	28	28	10	10
non-*var2csa*	4	4	12	1

**Significant surface labeling by VAR2CSA antibodies with MFI ratio >1.2.

a adhesion defined as binding ≥35 IE/mm^2^.

b binding level <35 IE/mm^2^.

### Adhesion phenotype of parasites is associated with parity and gestational age of women

Isolates from primigravidae bound on average to a higher level to CSPG than those from multigravidae (*P = 0.05*). Conversely, isolates from both primi- and multigravidae bound CD36 and ICAM-1 to similar levels (Table 5). Likewise, when the threshold of significant binding was applied, the analysis revealed a trend of parasites from primigravidae to adhere more frequently (OR = 3.2) to CSPG than those from multigravidae, although not strictly significant (*P = 0.11*), possibly due to a lack of power associated to our limited sample size. Although the affinity for CD36 was more advantageous among isolates from multigravidae with an unfavorable linear coefficient of -52.3 among isolates from primigravidae (Figure 2B), this relationship was not observed in our model of logistic regression analysis (OR = 0.64, *P = 0.6*) (Figure 2B). Regarding adhesion to ICAM-1, the logistic regression model failed to converge, due to numerical trouble.

The article "Dynamics in the Cytoadherence Phenotypes of Plasmodium falciparum Infected Erythrocytes Isolated during Pregnancy" was published in 2014. Journal: PLoS One.

**Table 5:** Parity and gestational age dependence of PAM-isolates binding properties.

	Linear regression		Logistic regression	
	Coefficient* (95% CI)	p	OR (95% CI)	p
Primigravidae and multigravidae^a^				
CSPG	118.1 (−3.01–239.38)	0.05	3.2 (0.76–13.24)	0.11
CD36	−52.36 (−193.09–88.37)	0.45	0.64 (0.12–3.48)	0.60
ICAM-1	0.93 (−5.46–7.33)	0.76	CD	
Early and late pregnancy^b^				
CSPG	128.74 (16.73–240.75)	0.03	2.13 (0.62–7.37)	0.23
CD36	−117.24 (−216.62–17.87)	0.02	0.14 (0.03–0.61)	0.01

*Difference in the mean of adhesion level between the considered and reference classes.

a Reference class: Multigravidae.

b Reference class: Early pregnancy (<16 weeks of gestation).

OR =  Odd ratio; CD =  convergence default.

To investigate whether gestational age is associated with a particular binding phenotype of isolates, a cut-off was made at 16 weeks of gestational age to define early (<16 weeks) and late pregnancy (>16 weeks). For ICAM-1 receptor, the mixed models failed to converge. Isolates from late pregnancy bound CSPG to a higher level than those from early pregnancy (*P = 0.03,* Table 4). The opposite was observed with CD36, with a lower binding level of late pregnancy parasites (*P = 0.02*). This lower ability of isolates from late pregnancy to bind CD36 was confirmed also by logistic regression analysis (OR = 0.14; *P = 0.01*). No association was observed between parasite density and binding phenotype of the isolates. In addition, when analysis was done according to the pregnancy outcome, such as the birth weight of the baby and the level of maternal hemoglobin, no relationship was observed with a particular adhesion pattern of IE.

## Discussion

The ability of *P. falciparum* IE to bind to CSA is the key factor that mediates placental sequestration and consequently the pathogenesis of malaria during pregnancy. Several studies have described the particular adhesion phenotype that characterizes parasites collected from women during pregnancy [3], [23], [25], [36], demonstrating evidence of a distinct binding ability to CSA shared by such isolates. Most of these studies have focused on isolates collected in late pregnancy [23], [25], [39], and observations have greatly helped formulate the hypothesis that the parasite ligand mediating adhesion to CSA would represent the main target for potential vaccine development against PAM. However, few studies have investigated the binding phenotypes of parasites infecting pregnant women early in pregnancy, their dynamics throughout pregnancy in relation to VAR2CSA expression, and whether pregnancy-related factors such as parity and gestational age can influence these phenotypes.

The article "Dynamics in the Cytoadherence Phenotypes of Plasmodium falciparum Infected Erythrocytes Isolated during Pregnancy" was published in 2014. Journal: PLoS One.

Recently, we have demonstrated that infection by CSA-binding isolates occurs in the first trimester of pregnancy [36]. Not all isolates collected at this stage of pregnancy bound to CSA. In this study, we collected and analyzed the parasites from peripheral blood of pregnant women at different times of pregnancy. In addition to CSA, we have now assessed which of the other receptors (CD36 and ICAM-1) are most commonly preferred by isolates collected throughout pregnancy and investigated whether infection by parasites with an adhesion pattern to these receptors in a particular timing of pregnancy could be associated with poor outcome. Variability in the binding phenotype of isolates was observed throughout pregnancy. Our data highlights the coexistence of parasites with several binding phenotypes in early pregnancy isolates. But, this diversity gradually tightens with gestational age in favor of the CSA binding phenotype. This finding points out the high risk of women infection by parasites with CSA-binding phenotype late in pregnancy, suggesting that isolates with adhesion pattern to other receptor are less involved in the pathogenesis of PAM requiring placental tropism.

However, adhesion to CSA was the most prevalent phenotype displayed by peripheral isolates from pregnant women compared to binding to either CD36 or ICAM-1. Generally, these isolates bound to CSA at higher levels compared to CD36 and ICAM-1. Although the placental tropism of CSA-binding parasites might explain this adhesion preference of the isolates, a possible role of the pre-existing immunity in these women, against CD36- and ICAM-1-binding parasites should be considered. This pre-existing immunity acquired from childhood mainly against CD36- and ICAM-1-binding parasites could be an important filter. As already described [20], [25], [39], interactions with ICAM-1 were observed with few isolates from pregnant women, while adhesion to CD36 was more frequently observed among isolates from multigravidae (28%) than those from primigravidae (20%). These observations clearly indicate that infections with parasites not adhering to CSA also occur during the pregnancy. Although the importance of these infections in the outcome of pregnancy is unknown, their characterization remains an open issue in the context of pregnancy success in malaria-endemic regions. Such infections are dependent on gestational age, occurring earlier in pregnancy and gradually decreasing with increasing gestational age. It is likely that the generalized immuno-modulation that occurs during pregnancy favors infections with *P. falciparum* regardless of the binding phenotype in primigravid women. The restriction of this phenotype to parasites with a preference for CSA occurs gradually as the placenta grows and becomes increasingly irrigated. It is quite plausible that interventions like IPTp also promote this phenotypic refining by increasing the fitness of placental parasites that will be more preferably selected in subsequent infections. On the other hand, non-CSA binding phenotypes seem to be more common in multigravidae, in whom immunity against CSA-binding parasites is well described [40], [41]. The re-emergence of infections with non-CSA binding parasites suggests better control of CSA-binding phenotypes via acquired immunity, thereby restoring the diversity of binding properties observed in non-pregnant individual. However, we did not observe a significant association between a particular adhesion phenotype of isolates and outcomes such as the maternal hemoglobin and birth weight of babies, probably due to the fact that all the infected pregnant women were systematically treated in this study.

The article "Dynamics in the Cytoadherence Phenotypes of Plasmodium falciparum Infected Erythrocytes Isolated during Pregnancy" was published in 2014. Journal: PLoS One.

Many studies have demonstrated the high susceptibility of women to PAM during the first pregnancy due to the lack of the protective immunity that is acquired following successive pregnancies [1], [15], [42]. In line with these reports, our data emphasize the high vulnerability of primigravid women to infection by parasites with a CSA-binding phenotype. This increased vulnerability suggests that these parasites that strongly adhere to CSA are those that cause the worst pregnancy outcomes, as supported by their high frequency in primigravidae, who are the most at risk of malaria consequences during pregnancy [1], [3], [42].

On the other hand, measurement of the transcription level of *var2csa* compared to other *var* genes were performed, and its expression as a protein on the surface of IE was assessed by use of specific anti-VAR2CSA antibodies. High transcription level of *var2csa* was observed among PAM-isolates, in agreement with prior reports that have identified this gene as being specifically highly transcribed in isolates from pregnant women. Although *var2csa* transcripts were detected in most isolates, infections with parasites that dominantly transcribed other *var* genes were observed. Most of these isolates preferentially bound to CD36 and/or ICAM-1. The binding preference to CSA was exclusively observed among isolates in which the transcription of *var2csa* was clearly dominant over that of the other *var* genes [43], [44]. Co-expression of multiple *var* genes, due to clonal phenotypic variation of parasites and to the multiplicity of infections, might explain the fact that some isolates were able to bind to more than one receptor.

The article "Dynamics in the Cytoadherence Phenotypes of Plasmodium falciparum Infected Erythrocytes Isolated during Pregnancy" was published in 2014. Journal: PLoS One.

The positive association between the surface expression of VAR2CSA and ability of IE to bind CSA supports previous reports indicating VAR2CSA is the main protein involved in this interaction. However, some few isolates did not bind CSA whilst simultaneously exhibiting both a marked predominant transcription of *var2csa* and a specific labeling of VAR2CSA on the IE surface. A plausible explanation might be that the immobilized receptor binding-assay does not fully reproduce the physiological conditions mediating *in vivo* interactions, due to differences in protein conformation and localization. However, previous studies have demonstrated a variable ability of placental isolates to bind CSA [3], [20]. Further investigations using cell-based methods under flow conditions are needed to better characterize these low CSA-binding isolates, and to assess whether other factors or proteins are involved in the CSA-binding process. Conversely, in some isolates that showed binding to CSA, predominant transcription of other *var* genes instead of *var2csa* was noted. The polyclonal nature of pregnant women infections may partially explain this observation. It is also possible that the dominant transcribed *var* genes in these isolates might encode for particular adhesion phenotype which was not explored in this study. However, a possible role of other non-VAR2CSA parasite proteins expressed on the surface of IE in the interaction with the CSA is not to be excluded. Further studies are still needed to make this clarification.

In summary, the data presented here are of capital importance in the context of VAR2CSA-based vaccine development. Actually the expression of VAR2CSA appears as the major feature shared by the *P. falciparum* parasites infecting pregnant women. These data suggest a major interest in VAR2CSA variants that express a strong adhesion ability to CSA as a critical aspect to be considered in the ongoing effort of vaccine development.
